The article "Green tea polyphenols alleviate early BBB damage during experimental focal cerebral ischemia through regulating tight junctions and PKCalpha signaling" was retracted in 2025. Reasons: duplicated images; overlap with earlier publications; unreliable data.

# Green tea polyphenols alleviate early BBB damage during experimental focal cerebral ischemia through regulating tight junctions and PKCalpha signaling

**DOI:** 10.1186/1472-6882-13-187

**Published:** 2013-07-21

**Authors:** Xiaobai Liu, Zhenhua Wang, Ping Wang, Bo Yu, Yunhui Liu, Yixue Xue

**Affiliations:** 1 The 96th Class, 7-year Program, China Medical University, Shenyang, Liaoning Province, 110001, People’s Republic of China; 2 Department of Neurobiology, College of Basic Medicine, China Medical University, Shenyang, Liaoning Province, 110001, People’s Republic of China; 3 Institute of Pathology and Pathophysiology, College of Basic Medicine, China Medical University, Shenyang, Liaoning Province, 110001, People’s Republic of China; 4 Department of Physiology, College of Basic Medicine, China Medical University, Shenyang, Liaoning Province, 110001, People’s Republic of China; 5 Department of Neurosurgery, Shengjing Affiliated Hospital of China Medical University, Shenyang, Liaoning Province, 110004, People’s Republic of China

**Keywords:** Green tea polyphenols, Cerebral ischemia, Blood–brain barrier, Tight junction, Protein kinase Cα

## Abstract

**Background:**

It has been supposed that green tea polyphenols (GTPs) have neuroprotective effects on brain damage after brain ischemia in animal experiments. Little is known regarding GTPs’ protective effects against the blood-brain barrier (BBB) disruption after ischemic stroke. We investigated the effects of GTPs on the expression of claudin-5, occludin, and ZO-1, and the corresponding cellular mechanisms involved in the early stage of cerebral ischemia.

**Methods:**

Male Wistar rats were subjected to a middle cerebral artery occlusion (MCAO) for 0, 30, 60, and 120 min. GTPs (400 mg/kg/day) or vehicle was administered by intragastric gavage twice a day for 30 days prior to MCAO. At different time points, the expression of claudin-5, occludin, ZO-1, and PKCα signaling pathway in microvessel fragments of cerebral ischemic tissue were evaluated.

**Results:**

GTPs reduced BBB permeability at 60 min and 120 min after ischemia as compared with the vehicle group. Transmission electron microscopy also revealed that GTPs could reverse the opening of tight junction (TJ) barrier at 60 min and 120 min after MACO. The decreased mRNA and protein expression levels of claudin-5, occludin, and ZO-1 in microvessel fragments of cerebral ischemic tissue were significantly prevented by treatment with GTPs at the same time points after ischemia in rats. Furthermore, GTPs could attenuate the increase in the expression levels of PKCα mRNA and protein caused by cerebral ischemia.

**Conclusions:**

These results demonstrate that GTPs may act as a potential neuroprotective agent against BBB damage at the early stage of focal cerebral ischemia through the regulation of TJ and PKCα signaling.

## Background

Ischemic brain damage is an extremely complex multi-factor, multi-level pathological process accompanied by structural and functional changes of blood-brain barrier (BBB) [1]. Many factors such as plasmin, gelatinases, free radicals, inflammatory factor, vasoactive substances, neuroglia and so on are involved in the changes of BBB permeability, resulting in a series of brain tissue damage during cerebral ischemia. Therefore, BBB damage plays an especially important role in the pathological changes of ischemia [2,3]. Since cerebral ischemia and BBB damage are closely correlated, approaches for protecting the BBB integrity and reducing BBB permeability could help to elucidate the underlying pathophysiological mechanism in brain ischemia, to guide treatment as well as to evaluate drug’s efficacy. A large amount of drugs have been screened to change the BBB permeability and to reduce the ischemic brain damage by acting on different therapeutic targets. Green tea is one of the world’s most popular beverages. Green tea polyphenols (GTPs) are the most important biologically active components of green tea, among which (-)-Epigallocatechin gallate (EGCG) is the main component and essential functional ingredient. EGCG has been proved to be a natural antioxidant and free radical scavenger [4]. Mounting evidence suggests that GTPs may help reducing neuronal damages in some neurodegenerative disorders such as Parkinson’s or Alzheimer’s diseases. Moreover, animal data demonstrated that EGCG improved focal ischemia/reperfusion-induced brain injury including the infarction volume, neurological deficit, etc by attenuating neuronal damage due to its potent anti-oxidant effects [5-7]. Our previous study observed the change of BBB permeability within 4 h after brain ischemia, and preliminarily confirmed the protective effects of GTPs on maintaining rat’s BBB integrity through inhibiting increased eaveolin-1 expression at the early stage of ischemia [8]. Thus, EGCG has a good prospect as a neuroprotective agent against brain ischemia due to its multi-targeted, multi-directional protective effects on the neuronal injury and BBB leakage.

BBB permeability is closely related to structural and functional alterations in the endothelial cells of cerebral microvessels and tight junctions (TJs) between adjacent cells. Caveolae-mediated internalization belongs to one of the classical transcellular pathways. We have previously demonstrated that the expression of caveolin-1, a marker protein of caveolae, significantly increased after middle cerebral artery occlusion (MCAO) in rats, associated with the increase in BBB permeability. And GTPs could decrease the mRNA and protein expression of caveolin-1, thus in turn decreased the BBB permeability [8]. Increased paracellular permeability following TJ barrier damage directly contributes to the developments of cerebral vasogenic edema, hemorrhagic transformation and increased mortality after ischemic stroke [9]. The TJ proteins claudin-5, occludin and ZO-1 contribute to the integrity of the BBB, and changes in their composition and expression are associated with increased vascular permeability [10,11]. We wondered whether GTPs could attenuate the BBB disruption by protecting the TJ barrier after brain ischemia. It is very necessary to clarify the neuroprotective effects of GTPs on cerebral ischemia, which has been the major purpose of this work.

Studies suggest that protein kinase Cα (PKCα) activation has a prominent role in the neuronal injury after brain ischemia. The occurrence of progressive ischemic neurodegeneration was accompanied by sustained increases in PKCα activity [12]. Recently, it has been reported that recombinant human angiopoietin1 could prevent BBB damage by inhibiting the expression of PKCα after focal cerebral ischemia/reperfusion in rats [13]. Moreover, PKCα serves as a regulator of brain endothelial paracellular permeability by alternating TJ proteins and F-actin filament reorganization [14]. GTPs have been reported to inhibit testosterone production in rat Leydig cells by inhibiting the PKA/PKC signaling pathways [15]. We aimed to observe the expression of PKCα in the ischemic brain tissue as early as 30 min after cerebral ischemia and the effect of GTPs on PKCα activity.

In the current study, we focused primarily on whether GTPs may reduce postischemic BBB damage by attenuating increased paracellular permeability in Wistar rats. To provide a more comprehensive insight into the neuroprotective effects of GTPs on early brain ischemia, we examined the changes in TJ morphology, the mRNA and protein expression levels of claudin-5, occludin, ZO-1 and PKCα in microvessel fragments of cerebral ischemic tissue within 2 h of ischemia following the prophylactic neuroprotective treatment of GTPs.

## Methods

### Animals and grouping

Adult male Wistar rats (250–300 g) were purchased from the Center of Experimental Animals, China Medical University. All experiments were performed in accordance with NIH Guidelines for the Care and Use of Laboratory Animals and approved by the Ethical Committee of Animal Experiments of the China Medical University. The animals were housed in laboratory cages maintained on a 12-h light-dark cycle, with free access to food and water throughout the study period. Mean arterial blood pressure was monitored and rectal temperature was maintained at 37°C during the surgery. Animals were randomly assigned to the control and GTPs groups. GTPs (400 mg/kg/day; Hangzhou Gosun Biotechnologies Co. Ltd, Hangzhou, China) were administered with intragastric gavage method twice a day for 30 day before surgery. Vehicle (saline) was given in the same way as mentioned above. Then experiments of each group were performed at four time points: 0, 30, 60 and 120 min after ischemia. After 30 d, all groups were performed surgery of middle cerebral artery occlusion (MCAO). The physiological parameters such as body weight, blood pressure or cerebral blood flow were maintained the same between the vehicle and GTPs-treated groups.

### Cerebral ischemia model

Focal cerebral ischemia was induced by MCAO at different time points in rats as described by Zea Longa [16]. Briefly, Rats were anesthetized with 10% chloral hydrate (350 mg/kg, i.p.). After a median incision of the neck skin, the left common, external, and internal carotid arteries were isolated. A nylon filament (diameter 0.26 mm) was inserted into the internal carotid artery via an incision in the common carotid artery and advanced until the rounded tip reached the origin to the left middle cerebral artery. To confirm proper MCAO, a laser-Doppler probe (Millwey, Axminste, UK) was fixed on the skull (1.5 mm posterior to the bregma and 5 mm from the midline on the left side) to measure local cortical blood flow in an area supplied by the middle cerebral artery during the operation. The successful occlusion was determined by a 30% decrease to baseline in local cortical blood flow. In the 0 min group, the rats underwent a similar surgical procedure but the left arteries were not occluded. The behavioral testing was assessed according to Zea Longa’s method. At different time points of ischemia, the rats were scored blindly on a five-point scale: 0 = normal; 1 = drags forepaw, twisting when lifted; 2 = circling spontaneously; 3 = falls; 4 = does not walk, comatose; 5 = dead [16]. The rats that obtained a score of 4–5 were excluded from the study.

### Evaluation of BBB permeability

Evans blue staining was performed to determine if GTPs treatment could alternate BBB permeability after a focal cerebral ischemia [17,18]. Briefly, 2% EB in saline (2 mg/kg) was injected intravenously 2 h before each expected time point. At expected time points after ischemia, rats were deeply anesthetized with 10% chloral hydrate and transcardially perfused with heparinized saline until colorless perfusion fluid was obtained from the right atrium. After decapitation, the hemispheres were separated along the sagittal suture. Both hemispheres were weighed and immersed into formamide (1 ml/100 mg) at 60°C for 24 h. The content of dye extracted from each brain was determined with a spectrophotometer (at 620 nm). The quantitative calculation of the dye content in the brain was based on the external standards dissolved in the same solvent.

### Transmission electron microscopy (TEM)

The postischemic Ultrastructural changes of TJ following prophylactic treatment with GTPs were examined using TEM. At expected time points after ischemia, the deeply anesthetized rats were perfused transcardially with 2.5% glutaraldehyde and 4% paraformaldehyde. The ischemic brain tissues were divided into some pieces of 1 mm^3^, fixed with 2.5% glutaraldehyde at 4°C. According to the standard procedures, semi-thin and ultra-thin sections were prepared and stained with uranyl acetate and lead citrate, and then samples were observed by TEM (JEM-1200EX, Japan).

### Reverse transcription-polymerase chain reaction (RT-PCR)

Cerebral microvessels were isolated from rat cortical gray matter for the analysis of TJs gene [19,20]. Isolated microvessels were routinely examined to confirm enrichment of microvessels. RT-PCR was used to investigate the mRNA expression of claudin-5, occludin, and ZO-1. Total RNA was isolated from the brain microvessel fragments of ischemic tissue using Trizol (Takara Biotechnology, Dalian, China) according to the manufacturer’s protocol. cDNA was generated from 1.0 μg of the total RNA from each sample with a reverse transcription kit by avian myeloblastosis virus reverse transcriptase. The applied PCR primers were as follows: claudin-5: (forward: 5′-CGGGCGTCCAGAGTTCA-3′, reverse: 5′- TTCAGCGGTGGTCGTCA-3′, 185 bp); occludin: (forward: 5′- TCGCTTCCTTGGTGA-3′, reverse: 5′-CAGAGGCGGTGACTTAT-3′, 593 bp); ZO-1: (forward: 5′- CTCGGGCATTATTCG -3′, reverse: 5′- CTCCAGGTTGACATTAGTT -3′, 817 bp); PKCα (forward: 5′ -GTGCCAAGTTTGCTGTT- 3′, reverse: 5′-CGCAGGTGTCGCATT-3′ 209 bp); ß-Actin: (forward: 5′-CATCTCTTGCTCGAAGTCCA-3′, reverse: 5′-CGCAGGTGTCGCATT-3′, 318 bp). PCR amplification was carried out for 30 cycles. β-Actin served as an internal control. PCR products were separated by electrophoresis on 1.5% agarose/TBE gels. Gels were photographed using the Chemi Imager 5500 gel image analysis instrument (AlPha InnCh). The integrated density value (IDV) of PCR product bands was calculated by computerized image analysis (Fluor Chen 2.0) and normalized with that of β-Actin.

### Immunohistochemistry

Immunohistochemical staining was used to determine the distribution and expression of claudin-5, occludin and ZO-1 in postischemic brain microvessels after pre-treatment with GTPs. Rat brains were post fixed in 4% paraformaldehyde for 24 h, and then immersed in 30% sucrose solution in phosphate-buffered saline for 24 h in both GTPs and control groups. Coronal sections at the level of the anterior commissure in the ischemic region were cut into 10-μm-thick pieces. The sections were incubated with anti-claudin-5 antibody (diluted 1:150; Santa Cruz Biotechnology), anti-occludin antibody (diluted 1:150; Santa Cruz Biotechnology), or anti-ZO-1 antibody (diluted 1:150, Zymed) at 4°C overnight, and then the remaining procedures conformed to the standard procedures. For semi-quantitative measurements of claudin-5, occludin and ZO-1 density, the sections were photographed and analyzed using a computer-assisted image analyzing system (MoticImages Advanced 3.2).

### Western blot assessment

Western blot was used to detect the protein expression of TJ associated proteins, PKCα in the ischemic cortex. Cerebral microvessel segments were obtained from rat cortical gray matter in the ischemic region as previously described [19,20]. Equal amounts of proteins were separated by 7.5% to 10% sodium dodecyl sulphate-polyacrylamide gels, electrophoretically transferred to nitrocellulose, and then stained overnight at 4°C respectively with anti-claudin-5 antibody (diluted 1:400; Santa Cruz Biotechnology), anti-occludin antibody (diluted 1:400; Santa Cruz Biotechnology), anti-ZO-1 antibody(diluted 1:400; Santa Cruz Biotechnology), anti-PKCα (diluted 1:400, Bioworld Technology, Inc.). After the protein was incubated with secondary antibody conjugated with horseradish peroxidase (diluted 1:3000; Santa Cruz Biotechnology) for 1 h at room temperature, enhanced chemiluminescence analysis (ECL kit, Santa Cruz Biotechnology) was performed to determine the immunoreactive bands. The protein bands were scanned with Chemi Imager 5500 V2.03 software, and the IDV were calculated using a computerized image analysis system (Fluor Chen 2.0) and normalized with that of β-Actin.

### Determination of PKCα activity

Cytosolic and membrane fractions of ischemic tissue were separated according to the procedure to evaluate the translocation of PKC [21]. And then, PKC activity of cytosolic and membrane fraction was measured. The following PKC assay was performed according to the manufacturer’s suggestions: colorimetric PKC assay (PepTag; Promega, Madison, WI) and specific PKCα assay (PKCα KinEASETM FP fluorescein green assay, Upstate) [14]. The PKC translocation was calculated for each group by the corresponding membrane-to-cytosol ratio.

### Statistical analysis

All data are presented as the means ± SD. Differences among multiple groups were statistically analyzed using one-way ANOVA. Two sample T-tests with Bonferroni’s correction were applied to test differences between groups. Statistical significance was assumed if *P* value was less than 0.05.

## Results

### GTPs attenuated BBB disruption after focal ischemia

The effects of GTPs on BBB permeability within 120 min after ischemia were evaluated with Evans blue staining. Increased Evans blue signal was detected in the ischemic hemispheres at 60 and 120 min after ischemia, whereas no staining could be observed in the 0 and 30 min ischemic groups. As shown in Figure 1, the content of Evans blue increased significantly at 60 and 120 min after ischemia in the saline-treated group as compared with the 0 min group (*P* < 0.01). There was no significant change in the Evans blue content of the ischemia between 30 min and 0 min group (*P* > 0.05). In the GTPs-treated groups, the exudation of Evans blue decreased significantly compared with the vehicle group at the time points of 60 min and 120 min after ischemia (*P* < 0.01). Evans blue staining results indicated that the increased BBB permeability could be attenuated by GTPs pre-treatment at the early stage of brain ischemia.

**Figure 1:** **Effects of GTPs on BBB permeability at the early stage of cerebral ischemia were assessed by Evans blue dye leakage.** Experiment groups are saline-treated (vehicle) groups and GTPs-treated groups at the time points of 0, 30, 60, and 120 min after ischemia, respectively. **(A)** representative images of brain sections in the groups of ischemia and GTPs-treated groups of ischemia at 120 min. **(B)** Evans blue content is expressed as a fold increase relative to the vehicle group of ischemia at 0 min. Data are given as the means ± SD (n = 8, each). ^**^P < 0.01 vs. vehicle group of ischemia 0 min. ^##^*P* < 0.01 vs. vehicle group at the same time points.

### GTPs altered the postischemic changes in TJ morphology

The results of TEM have qualitatively shown the changes in the integrity of the TJ barrier after GTPs treatment. In the vehicle and GTPs groups at 0 and 30 min, TJ lay in the plasma membrane of adjacent brain microvascular endothelial cells (BMECs) and sealed the intercellular cleft, appearing as a series of electron-dense zones (Figure 2A1, A2, B1, B2), whereas intercellular cleft was clearly recognized between adjacent endothelial cells in the vehicle groups at 60 and 120 min after ischemia (Figure 2A3, A4). In GTPs-treated groups, the reverse of TJ opening after ischemia was observed at 60 and 120 min after ischemia (Figure 2B3, B4), indicating that GTPs might repair the postischemic TJ integrity.

**Figure 2:** **The postischemic ultra structure of TJ after GTPs administration was examined by TEM.** Representative graphs of the following groups: **A1**–**A4**, the vehicle group at 0, 30, 60, and 120 min after ischemia; **B1**–**B4**, the GTPs group at 0, 30, 60, and 120 min after ischemia, respectively. Graphs **(A1**, **A2**, **B1**, **B2**, **B3**, **B4)** show that TJ barrier was intact. Graphs **(A3**, **A4)** display an increase in the gap at TJ. Arrows show TJ. Scale bars = 400 nm.

### GTPs changed the mRNA and protein expression of claudin-5, occludin, and ZO-1 following cerebral ischemia

To investigate the effects of GTPs on BBB disruption after brain ischemia, RT-PCR, immunohistochemistry and western blot were undertaken to determine the mRNA and protein expression of claudin-5, occludin, and ZO-1. As shown in Figure 3(A-D), RT-PCR results showed that the mRNA expression levels of claudin-5, occludin, and ZO-1 significantly decreased in cerebral microvessels in vehicle groups at 60 and 120 min after ischemia compared with that of 0 min group (*P* < 0.01). There was no significant difference in the expression of claudin-5, occludin, and ZO-1 between the vehicle groups at 0 min and 30 min, respectively (*P* > 0.05). The mRNA expression of claudin-5, occludin and ZO-1 was significantly promoted in the GTPs-treated groups at 60 and 120 min after ischemia compared with the vehicle groups at the same time points, respectively (*P* < 0.05, *P* < 0.01). There was no significant difference in the mRNA expression of claudin-5, occludin, and ZO-1 between the vehicle groups and the GTPs-treated groups at 0 and 30 min after ischemia, respectively (*P* > 0.05).

**Figure 3:** **Effects of GTPs on the expression of claudin-5, occludin, ZO-1, and PKCα mRNA at the early stage of brain ischemia were determined by RT-PCR. (A)** M, DNA ladder; V0–V120, 0, 30, 60, and 120 min after ischemia in the vehicle group; G0–G120, 0, 30, 60, and 120 min after ischemia in the GTPs-treated group. The mRNA levels of the gene expression were normalized to those of β-Actin as an endogenous reference. **(B**-**E)** IDV of claudin-5, occludin, ZO-1, and PKCα is expressed as a fold reduction or a fold increase relative to the vehicle group of ischemia 0 min. Data represent the means ± SD (n = 6, each). ** *P* < 0.01 vs. vehicle group of ischemia at 0 min. ^#^*P* < 0.05, ^##^*P* < 0.01 vs. vehicle group at the same time points.

The immunohistochemistry results revealed that the staining of claudin-5, occludin and ZO-1 was continuously, sharply, perfectly located in the cerebral microvessels of vehicle groups at 0 and 30 min. Loss of continuity in the distribution and attenuated expression of these three TJ associated proteins were observed in the vehicle groups at 60 and 120 min after ischemia. Moreover, the mean optical density values of claudin-5, occludin and ZO-1 were significantly decreased in the vehicle groups at 60 and 120 min after ischemia compared with those of the vehicle group at 0 min (*P* < 0.01). Claudin-5, occludin, and ZO-1 still presented a perfect localization and normal expression in the cerebral vascular structures in the GTPs-treated groups at 0 and 30 min after ischemia. The mean optical density values of claudin-5, occludin, and ZO-1 in the GTPs-treated groups at 60 and 120 min were significantly increased compared with those at the same time points, respectively (*P* < 0.01), indicating that GTP pre-treatment could protect the integrity of the BBB TJ barrier (Figure 4).

**Figure 4:** **Effects of GTPs on the distribution and expression of claudin-5, occludin, and ZO-1 in ischemic cerebral microvessels were analyzed by immunohistochemistry at 0, 30, 60 and 120 min after ischemia.** Representative immunohistochemistry stained graphs of claudin-5 **(A, C, E, G)**, occludin **(I, K, M, O)**, and ZO-1 **(Q, S, U, W)** at 0, 30, 60, and 120 min after ischemia in the vehicle group; graphs of claudin-5 **(B, D, F, H)**, occludin **(J, L, N, P)**, and ZO-1 **(R, T, V, X)** at 0, 30, 60, and 120 min after ischemia in the GTPs-treated group. Arrows show cerebral microvessels. Scale bar = 10 μm.

Western blot was performed to further investigate the protective effects of GTPs on the TJ barrier at the early stage of cerebral ischemia. In concordance with our RT-PCR and immunohistochemical staining results, the western blot results also verified that the expression of claudin-5, occludin, and ZO-1 proteins were significantly attenuated at 60 min and 120 min after ischemia compared with those at 0 min in the vehicle groups, respectively (*P* < 0.01). Accordingly, the expression of claudin-5, occludin, and ZO-1 proteins were significantly recovered at 60 and 120 min in the GTP-treated groups compared with those in the vehicle group at the same time points, respectively (*P* < 0.05, *P* < 0.01). Therefore, the expression of TJ associated proteins was promoted by GTPs pre-treatment, which indicated the protective effects of GTPs against the ischemic BBB leakage (Figure 5A-D).

**Figure 5:** **Effects of GTPs on the protein expression levels of claudin-5, occludin, ZO-1, and PKCα in ischemic cerebral microvessels after cerebral ischemia were determined by western blot. (A)** The lanes are the following groups: V0–V120, 0, 30, 60, and 120 min after ischemia in the vehicle group; G0–G120, 0, 30, 60, and 120 min after ischemia in the GTPs-treated group. β-Actin served as a internal control. IDVs of claudin-5 **(B)**, occludin **(C)**, ZO-1 **(D)** and PKCα **(E)** are expressed as a fold reduction or a fold increase relative to the vehicle group of ischemia at 0 min. Data represent the means ± SD (n = 6, each). ** *P* < 0.01 vs. vehicle group of ischemia 0 min. ^#^*P* < 0.05, ^##^*P* < 0.01 vs. vehicle group at the same time points.

### GTPs reduced the increased activity and expression of PKCα after Cerebral Ischemia

It has been reported that PKCα expression was significantly elevated after cerebral ischemia-reperfusion [13]. We further investigated the changes of PKCα expression and the effects of GTPs on PKCα pathway at the early stage of brain ischemia. As shown in Figure 3A, E, PKCα mRNA expression was significantly up-regulated at 60 min and 120 min after ischemia as compared with 0 min in the vehicle groups (*P* < 0.01). The mRNA expression levels of PKCα were significantly decreased at 60 and 120 min after ischemia in the GTPs-treated group compared with those in the vehicle group at the same time points, respectively (*P* < 0.01). The western blot and specific PKCα translocation assay data showed a similar tendency with the RT-PCR results. Membrane-to-cytosol ratio of PKCα activity and protein expression were also significantly attenuated by GTPs at the same time points after ischemia (Figure 5A, E; Figure 6, *P* < 0.01). These results revealed that GTP administration could attenuate the increased activity and expression of PKCα at the early stage of cerebral ischemia.

**Figure 6:** **Effects of GTPs on plasma membrane translocation of PKCα at the early stage of brain ischemia were determined by specific PKCα assay.** Quantification of PKC activity in the membrane-to-cytosol ratio was expressed as a fold increase relative to the vehicle group of ischemia at 0 min. Data represent the means ± SD (n = 6, each). ^**^P < 0.01 vs. vehicle group of ischemia 0 min. ^##^*P* < 0.01 vs. vehicle group at the same time points.

## Discussion

The present study demonstrated that the prophylactic neuroprotective treatment with GTPs modulated the postischemic changes of TJ barrier and PKCα signaling in rat models of MCAO. GTPs significantly reduced the BBB permeability after cerebral ischemia within 120 min. The mRNA and protein expression of TJ-associated proteins claudin-5, occludin, and ZO-1 were significantly decreased at the early stage of ischemia. Accordingly, the opening of the TJ barrier was observed by ETM. Whereas, GTPs significantly prevented the reduction of claudin-5, occludin, and ZO-1 expression at the time points of 60 and 120 min after ischemia. The PKCα expression was also found to be increased significantly and could be blocked by GTPs pre-treatment at 60 and 120 min after ischemia. These results demonstrated that increased paracellular permeability was also involved in the BBB disruption during the early stage of cerebral ischemia, and GTPs might protect BBB TJ integrity by enhancing the expressions of claudin-5, occludin, and ZO-1 and inhibiting PKCα expression.

Ischemic cerebrovascular disease has been paid more attention to by neurologists because of its high disability and death rate as well as refractory neuron damage. The aims of neuroprotective treatment for ischemic stroke are to prevent the harmful physiopathologic changes, to further reduce neuron damage, to improve survival rate and status and to decrease the rate of disability [22]. The concept of neurovascular unit emphasizes that the overall protection of the brain after ischemic stroke also includes vessels and glial cells apart from the neuron damage [23]. Recently, plant polyphenols have shown some promising effects as potent free radical scavengers in treating stroke. It has been reported that EGCG reduced the infarction volume, the neurological deficit total score, the level of malondialdehyde and the ratio of oxidized/total glutathione in rat transient focal ischemia models with 24-h reperfusion following 2-h occlusion of the middle cerebral artery [7]. Moreover, EGCG was also reported to protect against neuronal damage and brain edema after unilateral cerebral ischemia in gerbils [24]. During the early stage of cerebral ischemia, it was thought that the BBB disruption and glial cells damage played a more important role than neuron damage in the pathogenesis of cerebral ischemia. We have preliminary found that GTPs could protect BBB damage from 1 h after ischemia [8]. Since GTPs may protect against ischemic brain injury concurrently through the different mechanism, we further investigated the potential protective mechanism of GTPs on BBB damage in rat models of early focal cerebral ischemia.

The structural and functional changes and damage of BBB after cerebral ischemia could be the initiating factors for a series of irreversible neurodegenerative disorders [25]. Generally, increased vascular permeability determined by EB extravasation was observed within 1-2 h after cerebral ischemia, and remained until 24 h in the process of ischemia [26]. There have been reports demonstrating that early BBB permeability was increased from 30 min after MCAO [27]. Whereas, barrier damage determined by HRP permeability appeared immediately at the 2nd min after complete cerebral ischemia induced by cardiac arrest in the rat [28]. In this study, BBB opening appeared at 60 min following cerebral ischemia induced by MCAO, and GTPs might significantly attenuate this early BBB disturbance. The results were consistent with our previous report [8], reinforcing the notion that GTPs administration has a protective effect on early BBB permeability alterations after ischemic insult.

BBB disturbances during cerebral ischemia are associated with the multifactorial impairment such as TJ opening between BMECs, increased expression of AQP4 and matrix metallo proteinases (MMPs), free radical generation and so on [29,30]. Disruption of TJ barrier integrity and subsequent increase of paracellular permeability are major contributors to the pathogenesis of BBB damage in ischemic stroke [30]. Our TEM results showed an increase in the gap at TJ from 60 min following MCAO, indicating that TJ barrier alterations participated in early BBB changes after cerebral ischemia in rats. Claudin-5, occludin, and ZO-1 are the major structural proteins of the TJs, and the changes of their expression are closely related to the paracellular permeability of BBB and brain edema [11,31]. Previously, we confirmed that the expression levels of these TJ associated proteins were significantly decreased compared with the sham-operated group within 120 h of reperfusion in a time-dependent manner [32]. In this study, we focused on their expression during the early ischemia within 120 min. The RT-PCR, immunohistochemical staining and western blot results demonstrated that the expression of claudin-5, occludin, and ZO-1 has already decreased from 60 min after ischemia, which further verified the specific roles of these three TJ proteins in a focal cerebral ischemic insult.

As a natural beverage, the medical and health benefits of green tea are paid more and more attention to. GTPs, as a potent free radical scavenger and antioxidant, were reported to be used in the prevention and treatment of chronic diseases such as heart disease, various types of cancer and neurodegenerative diseases [33]. Previously, we first reported that a prophylactic treatment with GTPs for 30 d before MCAO could decrease the elevated transcelluar BBB permeability during the early brain ischemia by reducing the expression of caveolin-1 [8]. In this study, we investigated deeply the mechanism relating the protective effects of GTPs aganist early ischemic BBB damage. The results showed that the postischemic decreased expression of claudin-5, occludin, and ZO-1 was significantly ameliorated by GTPs pre-treatment. Collectively, preventive medication of GTPs could exhibit significant neuroprotection against early cerebral ischemia by elevating both transcelluar and paracelluar BBB permeability.

Numerous studies have demonstrated that PKCα might play an important role in the regulation of BBB permeability during the cerebral ischemia [14]. Our previous data demonstrated that PKCα expression in the ischemic brain microvessels was significantly increased at 12 h, 48 h and 7d after focal cerebral ischemia/reperfusion in rats, and the up-regulated expression of PKCα might be closely associated with the down-regulated expression of occludin and ZO-1 caused by ischemia/reperfusion injury [13]. Subsequent studies have demonstrated that the activity and expression levels of PKCα were up-regulated at 60 min and 120 min after ischemia. The time course was consistent with that of TJs changes, which heightened the speculation that the expression changes of PKCα were related to TJ alterations during brain ischemia. There are reports indicated that GTPs could inhibit PKCα signaling in several types of cells [15,34]. We have also characterized the effect of GTPs on the postischemic changes of PKCα. The up-regulation of membrane-to-cytosol ratio of PKCα activity and expression was alleviated by GTPs pre-treatment, suggesting that PKCα was possibly involved in the process of GTPs protection against early cerebral ischemia.

## Conclusions

In conclusion, we have reported for the first time that pre-treatment with GTPs alleviated MCAO-induced BBB damage by protecting the TJ barrier intact and inhibiting PKCα signaling in rats. The results have given another insight into the thinking that GTPs could be chosen as a potential multi-targeted neuroprotective agent in the treatment of early cerebral ischemia.

## Abbreviations

GTPs: Green tea polyphenols; BBB: Blood-brain barrier; MCAO: Middle cerebral artery occlusion; TJ: Tight junction; EGCG: Epigallocatechin gallate; MMPs: Matrix metallo proteinases.

## Competing interests

The authors declare that they have no conflicts of interest concerning this article.

## Authors’ contributions

XL carried out all of the experiments, drafted the manuscript and revising it. ZW drafted the manuscript and revising it. PW and BY performed the statistical analysis. YL and YX contributed to the design of the study, and revising the manuscript. All authors have read and approved the final manuscript.

## Pre-publication history

The pre-publication history for this paper can be accessed here:

http://www.biomedcentral.com/1472-6882/13/187/prepub
